The article "TCM Treatment and Drug Co-Occurrence Analysis of Psoriasis" was retracted in 2023. Reasons: unreliable results or conclusions; lack of ethics approval or compliance; missing or withdrawn patient consent; concerns about the data.

# TCM Treatment and Drug Co-Occurrence Analysis of Psoriasis

**DOI:** 10.1155/2022/4268681

**Published:** 2022-01-29

**Authors:** Li Lin, Suqing Yang, Qingsong Bai, Yuepeng An

**Affiliations:** ^1^School of Graduate, Heilongjiang University of Chinese Medicine, Harbin 150040, Heilongjiang, China; ^2^Department of Dermatology, First Affiliated Hospital, Heilongjiang University of Chinese Medicine, Harbin 150040, Heilongjiang, China

## Abstract

Psoriasis is a long-term immune-mediated disease. Patients with a long history and slow progress are more common, and its treatment is difficult. This study proposes to use traditional Chinese medicine to treat psoriasis. Through the follow-up of all participants for 12 and 24 weeks, a large number of comparative experiments effectively verify the effectiveness of the method proposed in this study. The research results of this study can provide some reference ideas for follow-up research.

## 1. Introduction

### 1.1. Psoriasis (Chart 1)

Approximately 1–3% of the world's population has some degree of psoriasis, which can be remitted and recur. Although a skin biopsy specimen's histological study may assist confirming the diagnosis, it is usually determined based on clinical symptoms alone [1]. Research shows that eventhough it is not life-threatening, the condition of having psoriasis may be severely debilitating and has substantial social and economic ramifications [2]. The biology of psoriasis is now well understood, and therapeutic advancements are helping even the most severely affected people. A considerable number of patients have a family history of disease, and some families have obvious genetic tendency. It is generally believed that about 30% of them have a family history. The incidence rate varies widely among different races. Psoriasis is a polygenic genetic disease with the interaction of genetic factors and environmental factors. The incidence of some HLA antigens in patients with this disease was significantly increased. Psoriasis may overlap with other diseases (such as rheumatoid arthritis and atopic dermatitis).

Eventhough it affects people of all ages, psoriasis manifests itself in two stages: the first happens in teens and young adults (between the ages of 16 and 22) and the second occurs in older people (at 57–60 years of age). Typically, the visible symptoms consist of circumscribed, thickened, scaly plaques that are pruritic and can be found on the elbows, knees, thighs, and buttocks as well as the scalp and areas of local trauma (Koebner's phenomenon). It is customary to measure the severity of involvement by using the psoriasis region and severity index, which consider factors such as the extent of the area involved, the redness, the thickness, and the scaling [3]. The plaques are characterized by a significantly thicker, horny layer (hyperkeratosis), and the dryness and cracking of this layer are responsible for much of the pain, itching, and inflammatory changes that result. On the psoriasis index, the maximum possible score is 72, and mild, moderate, and severe psoriasis are indicated by values of less than 10, between 10 and 50, and greater than 50, respectively. Plaques of psoriasis may naturally regress without leaving scars after a few weeks, months, or even years. Relapses are also prevalent, and by avoiding exacerbating variables, it is possible to lessen the frequency and severity of relapses in affected people [4]. These relapses are likely to occur in certain cases as a result of the activation of local wound-healing mechanisms in the body. Many scholars have confirmed that streptococcal infection is related to the onset and course of psoriasis from the aspects of humoral immunity (antistreptococcal group), cellular immunity (peripheral blood and skin lesion T cells), bacterial culture, and treatment. In patients with psoriasis, Staphylococcus aureus infection can aggravate skin lesions, which is related to the superantigen of Staphylococcus aureus exotoxin. The occurrence of this disease is related to virus. Although there is a certain relationship between viral (such as HIV virus) and fungal (such as *Malassezia*) infection, its exact mechanism has not been finally confirmed.

### 1.2. Symptoms of Psoriasis

The signs and symptoms of psoriasis may vary from person to person. Here are some examples of frequent indications and symptoms:

- The crimson flesh on the arms and legs is covered in large, silvery scales
- Scaling spots of varied sizes (often observed in youngsters)
- Dry, cracked, and itchy skin with the potential to bleed or itch. Itching, burning, or pain are all possible symptoms.
- Nails that are enlarged, pitted, or ridged swollen and stiff joints. The following formula was used to determine the sample size.

(1) $$\begin{array}{c} n=\frac{z_{2}\cdot p\cdot q}{d_{2}}, \end{array}$$

where *n* represents the sample size requested. The standard normal deviation is denoted by *z* (1.96). *p* represents the the estimated percentage of the target population who have the attributes being targeted. *q* = 1 − *p d* represents the statistical significance level (5%).

Psoriasis vulgaris is the most common type, with frequent acute onset. The typical manifestation is erythema with clear boundary and different shapes and sizes, surrounded by inflammatory erythema, slightly infiltrated and thickened. The surface is covered with multiple layers of silvery-white scales. The scales are easy to scrape off. After scraping, it is a light red and shiny translucent film, and small bleeding points can be seen when scraping the film. Skin lesions often occur in the head, sacrum, and lateral extension of the limbs. Some patients felt different degrees of pruritus.

According to the data in Table 1, the vast majority of 96% of patients had psoriasis vulgaris, 16% had pustular psoriasis, 0.7% had erythrodermic psoriasis, and 1.3% had psoriatic arthritis. Of the 11751 patients who had nonmissing disease activity data, 43.3% were in the active stage, 34.1% were stable, 15.3% were resolving, and 7.3% were remitting their symptoms.

## 2. Types of Psoriasis

In China and other countries, there exist different types of psoriasis, which have been occasionally treated by TCM.

### 2.1. Plaque Psoriasis

Plaque psoriasis is a persistent autoimmune disorder that affects the skin. It manifests itself on the skin as thick, red, and scaly areas of the skin (Figure 1). Plaque psoriasis can be an extremely itchy and unpleasant condition, especially in the early stages [5]. It can also be embarrassing, and it does not always respond to medical therapy as expected. It is occasionally mistaken as another skin ailment, such as dermatitis or eczema, and treated as such. Plaque psoriasis is characterized by regions of rough, red skin that are covered with silvery-white scales. This occurs as a result of the skin cells receiving a signal to make new skin cells at an excessively rapid rate [6]. They accumulate and shed in the form of scales and patches. Arthritis psoriasis is also known as psoriatic arthritis. Psoriatic patients have rheumatoid arthritis like joint damage at the same time, which can affect the joints of the whole body, but the lesions of the distal finger (toe) internode joints are the most characteristic. The affected joints are red, swollen, and painful, and the skin around the joints is often red and swollen. The joint symptoms are often aggravated or alleviated at the same time as the skin symptoms. The blood rheumatoid factor is negative.

In addition to causing red and silvery spots on the skin, this buildup of the skin also causes pain and inflammation. Scratching can result in abrasions, bleeding, and infection of the skin. Affected body parts include the elbows, knees, and scalp, which are among the most regularly observed. In these regions, the majority of people who suffer from plaque psoriasis will grow patches of the skin. However, some people will develop psoriasis patches on other parts of their bodies as well. The appearance of psoriasis patches on the body might be unpredictable in its spread. Some patches may be large enough to cover large areas of the body, while others may be a little larger than a dime in diameter.

Once a person has developed psoriasis, it may manifest itself in a variety of different ways and in different locations. The pubic area and armpits are frequently spared when it comes to plaque psoriasis, in contrast to inverse psoriasis.

As areas of plaque psoriasis heal, the position of the lesions may shift. During subsequent attacks, new patches may appear in other locations. Plaque psoriasis manifests itself differently in each individual. No two persons will have the same symptoms as one another.

This kind of medicine includes carboplatin and taccathitol. It has good curative effect on plaque psoriasis. Carpotriol cream, ointment, and lotion (for the head) are applied externally twice a day. It usually takes the effect within 8 weeks and will not be dependent after long-term use. The combination of this drug with glucocorticoid or UVB can improve the curative effect. It should be used with caution in patients with bone diseases, calcium metabolism disorders, and renal insufficiency, so as not to cause hypercalcemia.

Psoriasis can manifest itself as a range of nail lesions that are both distinct and ambiguous (Figure 2). Fingernails are more frequently affected than toenails (Figure 3), which is likely because fingernails develop more quickly.

As observed in this graph, there was no statistically significant difference in overall NAPSI scores between the left and right hands or between fingers with symmetrical lengths. NAPSI was greater for the thumb than for the other fingers, on the other hand. The forefinger, ring finger, and little finger all had higher NAPSI scores than a thumb (*p* 0.01) and forefinger (*p* 0.01), although the thumb (*p* 0.01) had lower NAPSI scores than all three (*p* 0.05, 0.05, and 0.0001) (Figures 4–6).

A variety of tests have determined that the response is either all-encompassing, restricted to the nails exclusively, or a hybrid of the two. Pitches are the small, sharp depressions on the nail's surface are the most common and immediately obvious symptom of a problem [7]. There are no differences in terms of size or depth between everything (Table 2). It is possible to distribute things at random or in transverse or short longitudinal lines that are parallel to one another. Small psoriatic foci develop in the apical matrix of these locations, producing parakeratosis and breaking of the proximal nail fold as it emerges. There is parakeratosis if the nail plate has an ivory-colored region in the proximal half [8]. As shown in Figure 4, It is possible to have one or many pits, and they may be associated with psoriasis or exist independently of the skin disorder. To have psoriasis, you need to have at least 10 craters on one of your nails.

The etiology of psoriasis includes genetic factors, immune factors, infection factors, endocrine factors, living habits, drug factors, environmental factors, and mental factors. Among them, endocrine factors and pregnancy can make the skin lesions disappear or reduce and can also aggravate the skin lesions. Thyroid diseases, diabetes, and other endocrine diseases have no obvious effect on the disease.

### 2.2. Treatment of Nail Psoriasis and Its Co-Occurrences

All therapies for nail psoriasis take a long time, since the nail is a slow epidermal attachment. The effectiveness of any treatment is seldom proved before 3–6 months, and it may take a year or more to get the greatest improvement feasible with a specific therapy [9]. As shown in Figure 5, to help patients visualize the therapeutic effects, photos taken before treatment is highly recommended. These photos should be presented to patients at all follow-up sessions [10]. As a result, before beginning treatment for nail psoriasis, patients should be screened for concomitant onychomycosis. A changed nail that remains despite appropriate treatment might be an indication of concomitant fungal infection. When onychomycosis is present, it might make it more difficult to treat the patient.

There are a variety of therapy options. As shown in Figure 6, some of the considerations that go into their decision-making include the degree of nail involvement and the impact on quality of life, as well as other conditions such as rheumatoid arthritis and other comorbidities [11]. Eventhough topical treatments for nail psoriasis are difficult to find, skin-cleansing systemic medicines work effectively for this condition [12]. There is a limited amount of topical medication that can reach the affected tissues because of the small nail fold and subungual hyperkeratosis in matrix lesions and nail bed psoriasis. Pits are the toughest wounds to cure, despite their subtle nature. An antipsoriatic topical therapeutic trial of three months is recommended (Figure 1). A shorter nail length increases the drug's ability to reach the psoriatic lesion. To treat nail bed psoriasis, the onycholytic nail must be cut over the infected nail bed. Drilling holes in the nail plate using mechanical burrs or ablative lasers improves nail penetration after filing or grinding. Laser ablation is a method used to analyze solid samples in inductively coupled plasma mass spectrometry. The laser used for laser shirt burning is a high-power, high repetition laser with large area sampling. In this way, the sampling uniformity is good and is not limited by the type of sample. Laser ablation mass spectrometry can be used to analyze small areas of samples.

### 2.3. Guttate Psoriasis

This subtype tends to affect youthful adults and children. It is frequently caused by a bacterial infection, such as strep throat. It is distinguished by tiny, drop-shaped, scaling sores on the torso, limbs, or legs.

### 2.4. Inverse Psoriasis

This primarily affects the groin, buttocks, and breast skin folds. Smooth areas of the red skin are caused by inverse psoriasis, which worsens with friction and sweating. This kind of psoriasis can be caused by fungal infections.

### 2.5. Psoriatic Arthritis

The disease is characterized by inflamed and aching joints, which are archetypal of arthritis symptoms. Sometimes, the symptoms of psoriasis in the joints are the first or only symptom or sign of the disease. There are times when only nail changes are visible. Psoriatic arthritis manifests itself in a variety of ways, ranging from moderate to severe, and can affect any joint. Stagnant joints can become stiffer as a result of this, and in the most severe cases, joint damage can become irreversible.

#### 2.5.1. Causes of Psoriasis

An issue with the immune system produces psoriasis, which causes the skin to regenerate at a quicker pace than normal. Plaque psoriasis is the most prevalent variety of psoriasis, and it is characterized by a rapid turnover of cells that results in scales and red patches of the skin. We still do not know exactly what it is that causes the immune system to malfunction [6]. Both genetics and environmental variables, according to the researchers, play a role. It is not contagious to have this illness.

The immune system is an important system for the body to perform immune response and immune function. It is composed of immune organs, immune cells, and immune molecules. The immune system has the function of identifying and eliminating antigenic foreign bodies, coordinating with other systems of the body, and jointly maintaining the stability of the internal environment and physiological balance.

#### 2.5.2. TCM Treatment and Drug Co-Occurrence of Plaque Psoriasis

In the Western world, the use of Chinese herbs to treat psoriasis is considered an alternative therapy because there is insufficient clinical evidence to support its effectiveness [13]. The traditional Chinese medicines Sheng Di Huang (also known as Qing Dia), Qian Cao Gin (also known as Qian Hua She Cao), and Bai Hua She Cao are considered mainstream options for the treatment of this skin condition among the billion or so people who live in China. When it comes to psoriasis treatment, traditional Chinese medicine (TCM) takes a completely different approach than when it comes to diagnosing and treating the condition in the West [14]. When it comes to traditional Chinese culture, the disease known as Bai Bi is supposed to be caused by “heat pathogens” which are responsible for the characteristic redness of the skin (Table 3).

According to some theories, blood “dryness” and “stagnation” are responsible for the itching, pain, and scaly plaque formation that characterize the autoimmune condition as the disease progresses.

Because traditional Chinese medicine is based primarily on impression and personal experience, the therapies prescribed by one practitioner may differ from another [15]. In contrast to Western treatment, traditional Chinese medicine therapies do not so much treat the sickness as they do correct the imbalances that cause situations such as heat, dryness, and stagnation.

TCM remedies are frequently combined and matched to target certain imbalances. As shown in Table 4, it would be more appropriate to employ herbs that “clear heat” in higher quantities than herbs that ease stagnation or dryness if blood heat is the primary concern in a given situation.

Qian Cao gin is the Chinese name for the herb common madder, which is also known as yarrow (*Rubix rubiae*). This herb is said to contain blood-cooling and antiproliferative effects, which may help to temper, if not prevent the growth of psoriasis plaques. It is also used to treat acne.

A Chinese herb known as Qing Dai (Indigo Naturalis) is considered to have great heat-clearing qualities, as well as antiproliferative and anti-inflammatory properties. Qing Dai is also known as Indigo Naturalis in the west.

#### 2.5.3. TCM Treatment

TCM, which is a system of ancient medical practice that differs from contemporary medicine in its substance, methodology, and philosophy, plays an essential part in the health maintenance of Asian peoples, and it is becoming more frequently adopted in countries around the Western world [16]. Despite their growing popularity, there are still some misconceptions about traditional medicines and the standards they must satisfy to be effective. In this area, we try to dispel some of the most common myths.

For the longest time, Asia's medical system has relied on traditional Chinese medicine (TCM) [1]. Traditional Chinese Medicine was developed after tens of thousands of years of empirical research and refining (TCM). Until English missionaries arrived in China during the early 1800s, it was the only medical specialty available in the country [17]. They brought modern medicine's medications, equipment, and practices with them.

### 2.6. Psoriasis Dosage

(2) $$\begin{array}{c} \text{RBW }=\frac{\text{ABT }\left(g\right)}{\text{IB }\left(g\right)}. \end{array}$$

RBW represents the relative body weight, ABT represents the absolute body weight, and IB represents the psoriasis patient body weight.

These doses were calculated for every psoriasis patient concerning their weight.

TCM comprises a wide range of techniques (chart 4) including herbal medicine and acupuncture that are familiar to Westerners as well as practices that are new to most Westerners such as cupping (hot cup therapy), Tuina (massage), and Qigong (burnt mugwort therapy). Traditional Chinese medicine (TCM) research is currently focused on understanding the mechanisms of action of these treatments [18, 19]. For the most part, this Nature Outlook will focus on herbal remedies as their efficacy is almost equivalent to that of current pharmaceuticals.

### 2.7. Acupuncture TCM as an Analysis of Psoriasis

Using small needles inserted through the skin, practitioners apply pressure to certain points on the body to stimulate healing. Studies have shown that acupuncture, whether real or fake, is equally effective, demonstrating that the placebo effect is at play. By altering brain regions involved in processing pain, acupuncture is thought to boost the body's generation of natural analgesics [20]. True acupuncture, according to the results of several studies, may be useful in treating chronic pain problems like osteoarthritis/knee pain and carpal tunnel syndrome as well as low back pain and neck discomfort. The frequency of tension headaches may be reduced, and migraine headaches may be prevented using this supplement. This is provided in Center for Chronic Disease and Hypertension Fact Sheet on Acupuncture (NCCIH) [21, 23].

### 2.8. Tai Chi TCM as an Analysis of Psoriasis

Postures, gentle motions, mental attention, breathing, and relaxation are part of a workout program [17]. Patients with Parkinson's disease, as well as the elderly and those who practice Tai Chi, may find it helpful with balance and stability. It has also been shown to help people with fibromyalgia and back pain, as well as enhance the quality of life and mood in those with heart failure. More information can be found about Tai Chi by going to the National Center for Chronic Disease and Hypertension's Tai Chi Fact Sheet.

### 2.9. Aspects of TCM an Analysis of Psoriasis

A wide range of medical illnesses has been researched using TCM medications, including stroke, heart disease, mental illness, and respiratory ailments (such as bronchitis and the common cold). About one out of every five Americans, according to the results of a national poll, uses Chinese herbal medications to treat a variety of medical ailments (Parker et al., 2016). It is impossible to draw firm conclusions about the value of many studies because they are of low quality.

## 3. Conclusion

Psoriasis is a condition that tends to reoccur. The recurrence pattern differs from patient to patient. Recurrences may be frequent and early for some people, whereas remission may be long-term and recurrences are few for others. Patients may need long-term maintenance therapy as a result. Psoriasis has a lengthy history of recurrent flare-ups. RCTs that have been done in the past have failed to yield insights into how to reduce recurrence. Research conducted in the real world, on the other hand, may provide more long-term results. The clinical efficacy of biological drugs for the treatment of psoriasis has been evaluated in previous articles using retrospective real-world registration studies. In China, however, there has been no real-world or registration study on TCM as a psoriasis therapy.

## Figures and Tables

**Figure 1:** The first onset of psoriasis in patients.

**Figure 2:** Plaque psoriasis infected skin. Nail psoriasis and its co-occurrences.

**Figure 3:** Comparison of nail psoriasis (NP) severity of different fingers of each hand (*n* = 126).

**Figure 4:** Nail psoriasis.

**Figure 5:** Gender psoriasis patients seeking TCM medication in China.

**Figure 6:** The approval of TCM as a treatment for drug co-occurrence of psoriasis in Europe.

**Table 1:** Comparison of lesion distribution and triggering factors between genders with psoriasis.

	Total *N* = 12031, *n* (% = *n*/*N*)	Male (*N*_1_ = 7206), *n*_1_ (% = *n*_1_/*N*_1_)	Female (*N*_2_ = 4825), *n*_2_ (% = *n*_2_/*N*_2_)	*P*

Triggering factors				
Season	7243 (60.2)	4388 (60.9)	2861 (59.3)	0.203
Stress	4151 (34.5)	2414 (33.5)	1790 (37.1)	<0.001
Smoking	626 (5.2)	533 (7.4)	92 (1.9)	<0.001
Alcohol	2214 (18.4)	1794 (24.9)	405 (8.4)	<0.001
Sphagitis	3296 (27.4)	1816 (25.2)	1486 (31.0)	<0.001
Lesions distribution				
Leg	9348 (77.7)	5355 (74)	3993 (83)	<0.001
Scalp	9024 (75.0)	5797 (80)	3227 (67)	<0.001
Elbow	8069 (67.1)	4757 (66)	3312 (69)	0.183
Thigh	8042 (66.8)	4558 (63)	3484 (72)	<0.001
Forearm	7620 (63.3)	4402 (61)	3218 (67)	<0.05
Back	7602 (63.2)	4173 (58)	3429 (71)	<0.001
Upper arm	7298 (60.7)	4104 (57)	3194 (66)	<0.001
Waist	6639 (55.2)	3719 (52)	2920 (61)	<0.001
Abdomen	6405 (53.2)	3442 (48)	2963 (61)	<0.001

**Table 2:** Disorder of nail with psoriasis.

Characteristics	*N* = 12031 (% = *n*/*N*)

Nail damage, *n* (%)	3592 (29.9)
Nail pitting	2167 (18)
Oil drops	1765 (14.7)
Subungual hyperkeratosis	1395 (11.6)
Longitudinal ridging of nails	1326 (11.0)
Onycholysis	856 (7.1)
Onychomadesis	300 (2.5)
Joint damages^a^, *n* (%)	740 (6.2)
Digital joints	406 (3.4)
Knee joint	356 (3.0)
Toe joint	190 (1.6)
Ankle joint	131 (1.1)
Elbow joint	114 (0.9)
Wrist joint	114 (0.9)
Vertebral column	94 (0.8)

**Table 3:** Clinical features and treatment of psoriasis by TCM.

Characteristics	No. of cases (%)

Total	*N* = 12031
Treatment history	
Systemic treatments	9600 (79.8)
TCM^a^	8661 (72.0)
Vitamin A derivatives	2604 (21.6)
Immune depressants	1297 (10.8)
Glucocorticoids	1577 (13.1)
Topical treatments	10787 (89.7)
Glucocorticoids	9113 (75.7)
Vitamin D3 analog	3634 (30.2)
Tazarotene	2976 (24.7)
TCM^a^	2802 (23.3)
Salicylic Acid	2295 (19.1)
Other therapy	2634 (21.9)
Photo therapy	2220 (18.5)

**Table 4:** A summary of the patient population.

Characteristics	*N* = 12031

Sex, *n* (%)	
Male	7206 (59.9)
Female	4825 (40.1)
Age, *y*	
Minimum	1
Maximum	86
Mean (SD)	39.42 (18.4)
Family history of psoriasis, *n* (%)	
Family history of psoriasis	2781 (23.1)
Relatives	*N* = 4995
First degree relatives	2323 (46.5)
Second degree relatives	1538 (30.8)
Third degree relatives	1134 (22.7)
History of smoking and alcohol, *n* (%)	
Smoking history	4023 (33.4)

## Data Availability

The data used to support the findings of this study are included within the article.
